The article "MRI Images-Based Evaluation of Efficacy of Neoadjuvant Chemotherapy for Breast Cancer and Its Effect on Depression and Immune Function of Patients" was published in 2022. Journal: Contrast Media Mol Imaging.

# MRI Images-Based Evaluation of Efficacy of Neoadjuvant Chemotherapy for Breast Cancer and Its Effect on Depression and Immune Function of Patients

**DOI:** 10.1155/2022/8685680

**Published:** 2022-09-05

**Authors:** Ying Nie, Yingjuan He, Jianzhi Wang, Hongjun Zhang, Junpeng Su

**Affiliations:** ^1^Department of Immune, Basic Medical College of Mudanjiang Medical University, Mudanjiang 157011, China; ^2^Department of Medical Psychology, School of Public Health of Mudanjiang Medical University, Mudanjiang 157011, China; ^3^Department of Sports Teaching and Research, Mudanjiang Medical University, Mudanjiang 157011, China

## Abstract

The aim of this study was to investigate the therapeutic value of neoadjuvant chemotherapy for breast cancer (BC) based on magnetic resonance imaging (MRI) and to evaluate its effect on depressive mood and immune function in patients. 70 female patients with BC who received neoadjuvant chemotherapy were selected for the experiment to comprehensively evaluate the MRI image findings, immune cell levels before and after chemotherapy, as well as the depression score and influencing factors of the patients during chemotherapy. The results showed that 49 patients (70%) responded to treatment, and MRI showed that the breast mass after chemotherapy was significantly reduced. 55 patients experienced depressive mood during chemotherapy, and the incidence of depression was 78.5%. Adverse symptoms such as pain, worry, sadness, vertigo, and nausea are important factors in the development of depression in patients. However, there were no significant changes in the levels of CD4+, CD8+, CD4+/CD8+, and killer cells before and after chemotherapy, and only B cells showed a significant decrease (9.78 ± 3.65% and 7.63 ± 3.65%) (*P* *<* 0.05). In summary, neoadjuvant chemotherapy can effectively shrink the breast mass and provide favorable conditions for subsequent surgery, and its clinical efficacy can be more accurately assessed by MRI. Neoadjuvant chemotherapy has little effect on the immune function of patients, but it will promote patients to experience depression. It provides a reference for the clinical treatment and prognosis of BC patients.

## 1. Introduction

Breast cancer (BC) is one of the most common malignancies in women, and its incidence is about 7–10% of various malignancies in the body. The incidence of BC is often genetically related [1], tends to occur in people aged 40–60 years, and usually occurs in the breast glandular epithelial tissue, and if not diagnosed and treated in time, it will seriously affect women's physical and mental health or even endanger life [2].

Magnetic resonance imaging (MRI) is the main examination method of BC, which has high sensitivity and noninvasive advantages for early BC [3]. Molybdenum target radiography is easy to operate, affordable, and highly specific and is widely used in clinical practice. However, some studies have pointed out that its ability to distinguish residual tumors after chemotherapy from interstitial fibrosis or hyalinization is not strong, and the size of residual lesions is often misestimated [4]. Ultrasound is noninvasive, nonradioactive, and can evaluate the changes before and after chemotherapy in terms of lesion size, shape, internal echoes, blood flow changes, and axillary lymph nodes, but there are some limitations in the efficacy of chemotherapy for simple microcalcification and large segmental, multinodular, or ill-defined masses [5]. In recent years, MRI has gradually become the main means to evaluate the efficacy of neoadjuvant chemotherapy for BC, and its advantages include high diagnostic sensitivity, identification of residual tissue and fibrosis and hyperplasia or necrosis caused by chemotherapy, and detection of multifocal and multicentric lesions. The early treatment of BC is mainly radical resection surgery, and after surgery, the follow-up adjuvant therapy can be determined according to the specific pathological type, clinical stage, and whether there are high-risk factors [6]. In recent years, neoadjuvant chemotherapy has become more and more widely used in clinical practice. It refers to the chemotherapy before surgery, which applies to the following conditions: patients with large tumors who are not suitable for direct surgery, creating surgical conditions by shrinking the tumor with neoadjuvant chemotherapy; for patients who do not want to accept total mastectomy, neoadjuvant chemotherapy can improve the breast-conserving surgery rate and retain part of the breast; some clinical studies have shown that the recurrence rate of some patients receiving neoadjuvant chemotherapy followed by surgery is lower than that of surgery followed by chemotherapy. According to their situation, these patients choose neoadjuvant chemotherapy as more appropriate [7, 8]. With the research and development of more new anticancer drugs, how to protect organ function to the greatest extent is a hot spot. Neoadjuvant chemotherapy can better locally control the tumor while breast-conserving and ensure the good quality of life of patients. In the future, it is expected to bring greater progress to the treatment of BC.

The article "MRI Images-Based Evaluation of Efficacy of Neoadjuvant Chemotherapy for Breast Cancer and Its Effect on Depression and Immune Function of Patients" was published in 2022. Journal: Contrast Media Mol Imaging.

Depression is a common psychological disease, with continuous and long-term depression as the main symptoms, which can also be manifested as mental retardation and decreased will activity [9]. Such negative emotions are common in patients with BC. The diagnosis of cancer will bring great psychological pressure on patients. During chemotherapy, drugs will cause certain adverse effects on human cells, and patients will have various clinical symptoms, such as nausea and vomiting, hair loss, allergy, and poor sleep quality. In addition, some patients have insufficient cognition or lack of confidence in chemotherapy, which will seriously affect their mental health of patients [10, 11]. In addition, long-term depression can bring additional negative effects on the physiological function of patients based on chemotherapy, reduce the resistance of tissues to cancer cells, further affect the effect of chemotherapy, and hinder the treatment process of patients [12, 13].

In the existing studies, there are few articles exploring the effect of neoadjuvant chemotherapy on depression and immune function in patients with BC. 70 female patients with BC who received neoadjuvant chemotherapy were selected as the study subjects. The clinical efficacy of neoadjuvant chemotherapy in BC and the effect on negative emotions and immune function of patients were innovatively explored by comprehensively evaluating their MRI image findings, immune cell levels, depression scores, and influencing factors, providing a theoretical reference for the clinical treatment and prognosis of patients with BC.

## 2. Materials and Methods

### 2.1. Subjects

Seventy female patients who received neoadjuvant chemotherapy from August 2019 to December 2020 were enrolled, with an age range of 27–56 years, with an average age of 38.78 ± 2.64 years. Patients and their family members agreed to sign an informed consent form. This study was approved by the ethics committee of the hospital.

Inclusion criteria were as follows: patients were diagnosed with BC by needle biopsy; the tumor was between 2 cm and 5 cm, accompanied by positive epidermal growth factor receptor 2 (HER-2); patients received at least 4 cycles of neoadjuvant chemotherapy; patients received MRI examination before and after chemotherapy and had sufficient MRI data; after neoadjuvant chemotherapy, patients received modified radical mastectomy or breast-conserving surgery; and the patient does not have any mental illness or disorder.

Exclusion criteria were as follows: male BC patients; secondary, inflammatory, and double BC patients; patients with metastasis or local recurrence; patients who are taking antidepressants or receiving psychotherapy; patients receiving endocrine therapy with chemotherapy; and patients with poor compliance and not cooperating with treatment.

### 2.2. Neoadjuvant Chemotherapy Regimens

Neoadjuvant chemotherapy regimens included four types. Anthracyclines: CAF, CEF, AC (C: cyclophosphamide; A: doxorubicin, E: epirubicin, F: fluorouracil); anthracyclines combined with taxanes: AC-T, EC-T, TAC, TEC (T: paclitaxel); and combined anti-HER-2 targeted therapy: tocilizumab; combined platinum drugs: cisplatin and lobaplatin. All patients received no less than 4 cycles of a neoadjuvant chemotherapy regimen.

The article "MRI Images-Based Evaluation of Efficacy of Neoadjuvant Chemotherapy for Breast Cancer and Its Effect on Depression and Immune Function of Patients" was published in 2022. Journal: Contrast Media Mol Imaging.

### 2.3. Breast MRI Examination and Image Processing

Patients were examined by a 3.0 T magnetic resonance imaging instrument. The patient was placed in the prone position, the breast was naturally suspended in the array coil, the parameters in line with the patients' condition were set, the horizontal and sagittal positioning scan of the breast was performed using a spin echo sequence, and a rapid inversion recovery sequence, with a slice thickness of 5 mm. Each patient received an intravenous contrast agent for an enhanced scan, and a dynamic enhancement curve was obtained (2 min).

The resulting data were processed using the processing software included in the Siemens magnetic resonance imaging system, and the breast mass area before and after treatment was delineated by two experienced professional imaging physicians, respectively, and if there were differences, the consensus was needed.

### 2.4. Immune Cell Testing

On the day before neoadjuvant chemotherapy and the second day after the end of all chemotherapy cycles, venous blood was drawn from the patients in a fasting state once and sent to the clinical laboratory. T cells (total B cells, CD4+, CD8+, and CD4+/CD8+) and natural killer cells (NK) were measured by CytoFLEX flow cytometry.

### 2.5. Evaluation Criteria for Neoadjuvant Chemotherapy

Response evaluation criteria in solid tumors [14] were referred, which were mainly based on single-path measurement. The evaluation criteria for target lesions were as follows: complete response (CR): all target lesions disappear completely, and all pathological lymph nodes (including target nodules and nontarget nodules) shrink to normal size (short diameter <1 cm); partial response (PR): ≥30% decrease in the sum of diameters of all measurable target lesions; progressive disease (PD): ≥20% increase in the minimum sum of diameters of all measured target lesions or the appearance of any new lesion; stable disease (SD): the sum of the longest diameters of all target lesions shrinks but does not reach PR or increases but does not reach PD.

Effective: CR and PR. Ineffective: SD and PD.

### 2.6. Observation Indicators

Hospital Depression Scale (HADS-D): it is widely used in clinical practice and consists of 7 items to assess depressive symptoms, each of which is scored as follows. 0, never; 1, occasional few days; 2, often; 3, almost every day. The total score is the sum of the scores of each item. The theoretical score is 0–21 points. The higher the score, the greater the likelihood of screening for depression.

The article "MRI Images-Based Evaluation of Efficacy of Neoadjuvant Chemotherapy for Breast Cancer and Its Effect on Depression and Immune Function of Patients" was published in 2022. Journal: Contrast Media Mol Imaging.

Patient Health Questionnaire (PHQ-9): it is a simple self-assessment questionnaire for depression, including 9 items, and the scores of each item are as follows. 0, never; 1, occasional few days; 2, often; 3, almost every day. The total score is the sum of the scores of each item. The theoretical score is 0–27 points. The higher the score, the greater the likelihood of screening for depression.

MD Anderson Symptom Inventory (MDASI): it is a simple and comprehensive self-rating scale that is widely used in the research field of cancer symptom management. It is mainly used to assess the intensity and frequency of core symptoms and the degree of interference of these symptoms with the patient's life, as well as to determine the relationship among various symptoms through the scoring of these symptoms and taking factor analysis. It aims to distinguish highly related symptoms from other symptoms and form a symptom cluster. Scores range from 0 to 10, with 0 being no such symptom and 10 being the most severe degree.

MRI findings and immune cell levels before and after neoadjuvant chemotherapy, depression scores of patients during chemotherapy, and resulting adverse reactions were observed and recorded.

### 2.7. Statistical Analysis

All experimental data were statistically analyzed, and scale data were analyzed by SPSS 24.0 software. Scale scores were expressed as mean ± standard deviation ($\bar{x}$±*s*), the frequency was used to analyze the degree distribution of depression, and the logistic multivariate regression model was used to analyze the effect of adverse symptoms on depression. Test level: *α*-0.05, two-sided test.

## 3. Results

### 3.1. Disease Data during Chemotherapy

Of the 70 female patients with BC, 61 patients were in the early and middle stages, the main pathological type was invasive ductal carcinoma, and half of the patients chose to be treated with anthracyclines combined with taxane chemotherapeutic drugs (Figure 1).

### 3.2. Clinical Response Evaluation of Neoadjuvant Chemotherapy

After 70 patients with BC completed neoadjuvant chemotherapy, the changes in the maximum diameter of the tumor before and after chemotherapy were assessed by MRI, and the clinical efficacy was assessed according to the response evaluation criteria for the treatment of solid tumors. 8 patients (11.4%) achieved CR, 41 patients (58.5%) achieved PR, 18 patients (25.7%) had SD, 3 patients (4%) had PD, and a total of 49 patients (70%) responded to treatment with CR + PR (Figure 2).

The article "MRI Images-Based Evaluation of Efficacy of Neoadjuvant Chemotherapy for Breast Cancer and Its Effect on Depression and Immune Function of Patients" was published in 2022. Journal: Contrast Media Mol Imaging.

### 3.3. MRI Image Evaluation of Response to Neoadjuvant Chemotherapy

A 60-year-old woman was admitted to the hospital with complaints of “a left breast mass found for more than 6 months.” MRI was performed to examine a hypoechoic nodule beside the left breast with blurred borders and irregular shapes. The diagnosis of BC (left) was confirmed by a needle pathological biopsy. After 6 cycles of neoadjuvant chemotherapy with AC-T, MRI was performed again, and the mass in the lower outer quadrant of the left breast shrank without a palpable mass in the breast (Figures 3 and 4).

### 3.4. Incidence of Depression in Patients during Neoadjuvant Chemotherapy

After 70 patients completed neoadjuvant chemotherapy, according to the HADS-D score and PHQ-9 score, 15 patients had no depression, 34 patients had mild depression, 17 patients had moderate depression, and 4 patients had severe depression. The incidence rate of depression was 78.5% (Figure 5). The mean HADS-D score was 8.46 ± 2.51 and PHQ-9 was 9.84 ± 2.55 in patients with mild depression; the mean HADS-D score was 11.15 ± 3.22 and PHQ-9 was 14.27 ± 3.41 in patients with moderate depression; and mean HADS-D score was 15.37 ± 4.62 and PHQ-9 was 18.87 ± 4.32 in patients with severe depression.

### 3.5. Effect of Patients' Symptoms on Depression during Neoadjuvant Chemotherapy

Patients experienced a variety of clinical symptoms during neoadjuvant chemotherapy, and the symptoms with a higher incidence included pain (93.2%), fatigue (92.8%), vertigo and nausea (92.1%), and sadness (90.4%) through the MDASI survey, and the symptoms with a higher score included sadness (4.15 ± 2.08 points), vertigo and nausea (4.07 ± 2.16 points), worry (3.87 ± 1.66 points), and pain (3.75 ± 1.43 points) (Table 1).

### 3.6. Logistic Multivariate Analysis Results

When the score of pain symptoms increased by one point, the risk of producing depressive mood was increased by 1.123 times, and the effect of pain symptoms on the occurrence of depressive mood in patients was statistically significant (*P* *<* 0.001), which was a risk factor for the occurrence of depression. Similarly, symptoms such as worry (*P* *<* 0.001), sadness (*P* = 0.002), and vertigo and nausea (*P* = 0.001) had a statistically significant effect on the generation of depressive mood in patients (Table 2).

### 3.7. Immune Cell Test Results of Patients before and after Neoadjuvant Chemotherapy

After the completion of neoadjuvant chemotherapy, CD4+ cells, CD8+ cells, CD4+/CD8+ cells, and NK cells were not significantly different from those before chemotherapy (*P* *>* 0.05), and only B cells (7.63 ± 3.65%) were significantly different from those before chemotherapy (9.78 ± 3.65%) (*P* *<* 0.05) (Figure 6).

The article "MRI Images-Based Evaluation of Efficacy of Neoadjuvant Chemotherapy for Breast Cancer and Its Effect on Depression and Immune Function of Patients" was published in 2022. Journal: Contrast Media Mol Imaging.

## 4. Discussion

BC is a malignant highly heterogeneous tumor that is a great threat to women, with some differences in histomorphology, immunophenotype, biological behavior, and treatment response, so early diagnosis and treatment are very important to prevent further development of the disease [15]. 70 patients with BC were selected and given a clinical neoadjuvant chemotherapy regimen, and the efficacy of chemotherapy was assessed based on MRI examination methods. Neoadjuvant chemotherapy specifically refers to preoperative chemotherapy. Its advantages include killing small metastases hidden in distant organs, so that tumor descent is conducive to the implementation of surgery and reducing the tumor to carry out breast-conserving surgery [16]. It can also observe the sensitivity of patients to chemotherapy drugs, which is helpful for doctors to adjust the treatment plan in time [17]. MRI has a high resolution for soft tissue and the sensitivity of breast MRI is higher than that of X-ray. It can observe the mass in three dimensions and not only provide the morphological characteristics of the lesion but also provide the hemodynamic status when dynamic enhancement is used. Therefore, it is widely used in the early diagnosis of BC. After 70 patients completed neoadjuvant chemotherapy, the clinical efficacy was assessed by MRI images as well as the response evaluation criteria for the treatment of solid tumors, and 49 patients responded to treatment, with a treatment response rate of 70%. Moreover, with the MRI image data of typical patients as an example, hypoechoic nodules could be detected beside the breast of patients before chemotherapy, with unclear boundaries and masses in the breast. MRI after neoadjuvant chemotherapy showed the masses in the lower outer quadrant of the breast shrank and no palpable masses. This is consistent with the study results of Takada and Toi [18]. The specific regimen of neoadjuvant chemotherapy needs to be developed according to the pathological type, clinical stage, physical condition, and other factors, shrinking and downstaging the tumor, facilitating the adoption of breast-conserving surgery, helping the patient eliminate potential subclinical lesions, and creating surgical conditions for patients with locally advanced disease. Hofmann et al. [19] also pointed out that MRI examination has a very high sensitivity for detecting breast lesions, and arbitrary three-dimensional imaging can make the lesion localization more accurate and more intuitive, providing a reliable basis for the staging of BC and detailed information for the development of treatment plans.

The article "MRI Images-Based Evaluation of Efficacy of Neoadjuvant Chemotherapy for Breast Cancer and Its Effect on Depression and Immune Function of Patients" was published in 2022. Journal: Contrast Media Mol Imaging.

However, most patients have insufficient awareness of neoadjuvant chemotherapy and lack confidence in the treatment, combined with a series of adverse reactions during chemotherapy, which can prompt patients to experience negative emotions. During chemotherapy, the body's antitumor immune mechanism is inevitably affected, causing some impact on the patient's immune cells and reducing the patient's immune function [20]. The HADS-D score, PHQ-9 score, and MDASI scale were used to investigate the patients during chemotherapy. The results showed that 55 of 70 patients had different degrees of depression, and the incidence of depression was 78.5%. The symptoms with higher incidence were pain, fatigue, vertigo, nausea, and sadness, and the symptoms with a higher score were sadness, vertigo and nausea, worry, and pain. By logistic multivariate regression model analysis, for each point increase in the score of pain, the risk of depression increased by 1.123 times. Worry, sadness, and vertigo and nausea can affect the occurrence of depression to a greater extent. Nakamura et al. [21] also had the same conclusion that while chemotherapy kills cancer cells, it also damages normal body cells, and the ensuing adverse reactions will cause negative emotions such as depression and anxiety in patients, affecting the compliance of treatment as well as the quality of life of patients. However, by detecting the level of immune cells in patients, there was no significant change in CD4+ cells, CD8+ cells, CD4+/CD8+ cells, and NK cells in patients before and after chemotherapy, and only the level of B cells (7.63 ± 3.65%) was significantly lower than those before chemotherapy (9.78 ± 3.65%) (*P* *<* 0.05). This may be due to the weak involvement of B cells in the process of tumor immunity and the strong killing effect of chemotherapeutic drugs on them.

## 5. Conclusion

The aim of this study was to evaluate the efficacy of neoadjuvant chemotherapy in patients with BC by MRI and to explore the effect of chemotherapy on depression and immune function. The results showed that neoadjuvant chemotherapy could shrink the breast mass and reduce the clinical stage, providing conditions for breast-conserving surgery. Chemotherapy largely affects patients to develop depressive moods and has little effect on immune function. The shortcomings are that the study subjects came from the same hospital, lacked representativeness, and only investigated the adverse symptoms of a certain chemotherapy cycle, and the investigation was not comprehensive enough. In the future, the experimental protocol will be improved to explore this topic in more depth.

The article "MRI Images-Based Evaluation of Efficacy of Neoadjuvant Chemotherapy for Breast Cancer and Its Effect on Depression and Immune Function of Patients" was published in 2022. Journal: Contrast Media Mol Imaging.

## Figures and Tables

**Figure 1:** Disease data of patients during chemotherapy. (a) Age. (b) Pathological type. (c) Clinical stage. (d) Chemotherapy regimen.

**Figure 2:** Clinical response assessment of neoadjuvant chemotherapy. (a) Number of patients with each rating. (b) Percentage of patients with each rating.

**Figure 3:** MRI images of the patient before neoadjuvant chemotherapy. (a)-(b) Horizontal images. (c)-(d) Sagittal images. Red areas are breast masses.

**Figure 4:** MRI images of the patient after neoadjuvant chemotherapy. (a)-(b) Horizontal images. (c)-(d) Sagittal images. Blue areas are breast masses.

**Figure 5:** Incidence of depression in patients during neoadjuvant chemotherapy. (a) Patient's depression. (b) HADS-D score. (c) PHQ-9 score.

**Figure 6:** Immune cell test results of patients before and after neoadjuvant chemotherapy. ^*∗*^B cells after chemotherapy are significantly different from those before chemotherapy (*P* < 0.05).

**Table 1:** MDASI assessment of patients during neoadjuvant chemotherapy.

Symptoms	Number of occurrences (times)	Percentage (%)	Score range (points)	Scoring ($\bar{x}$±*s*)
Pain	198	93.2	0–10	3.75 ± 1.43
Fatigue	187	92.8	0–10	3.62 ± 1.57
Vertigo and nausea	182	92.1	0–10	4.07 ± 2.16
Sadness	175	90.4	0–10	4.15 ± 2.08
Worry	170	87.6	0–10	3.87 ± 1.66
Tired	166	85.7	0–10	3.35 ± 1.69
Memory disorder	164	85.1	0–10	2.82 ± 1.45
Rapid breathing	159	83.9	0–10	3.58 ± 1.22
Dry mouth	152	82.8	0–10	2.67 ± 1.72
Sleep disturbance	148	81.6	0–10	3.15 ± 2.76
Palsy/sore and numb	136	75.4	0–10	2.83 ± 2.37

**Table 2:** Logistic multivariate analysis results.

Influencing factors	Regression coefficient	Standard error	Statistical quantity	*P*	Odds ratio	95% confidence interval
Pain	1.123	0.252	18.532	≺0.001	2.785	(1.663, 4.285)
Vertigo and nausea	0.653	0.173	10.638	0.001	1.746	(1.347, 2.402)
Sadness	0.784	0.189	9.368	0.002	1.843	(1.328, 2.682)
Worry	1.086	0.231	19.734	＜0.001	2.804	(1.705, 4.312)

## Data Availability

The data used to support the findings of this study are available from the corresponding author upon request.
